# Association between preventable risk factors and metabolic syndrome

**DOI:** 10.1515/med-2021-0397

**Published:** 2022-02-21

**Authors:** Hamoud A. Al Shehri, Abdulrahman K. Al Asmari, Haseeb A. Khan, Saud Al Omani, Saeed G. Kadasah, Ghaleb B. Horaib, Ahmed Al Buraidi, Abdullah A. Al Sharif, Fayez S. Mohammed, Rajamohamed Abbasmanthiri, Nasreddien M. Osman

**Affiliations:** Medical Service Department (MSD), Adult Cardiology, Prince Sultan Cardiac Center, Ministry of Defence, Riyadh, Saudi Arabia; Medical Service Department (MSD), Scientific Research Center, Ministry of Defence, P.O. Box: 22454, Riyadh 11495, Saudi Arabia; Department of Biochemistry, College of Science, King Saud University, Riyadh 11451, Saudi Arabia; Department of Surgery, Prince Sultan Military Medical City, Medical Service Department (MSD), Ministry of Defence, Riyadh, Saudi Arabia; Department of Psychiatry, Prince Sultan Military Medical City, Medical Service Department (MSD), Ministry of Defence, Riyadh, Saudi Arabia; Dermatology Department, Medical Service Department (MSD), Ministry of Defence, Riyadh, Saudi Arabia; Department of ENT, Prince Sultan Military Medical City, Medical Service Department (MSD), Ministry of Defence, Riyadh, Saudi Arabia; Department of Dentistry, Prince Sultan Military Medical City, Medical Service Department (MSD), Ministry of Defence, Riyadh, Saudi Arabia; Department of Radiology, Prince Sultan Military College of Health Science, Dhahran, Saudi Arabia

**Keywords:** metabolic syndrome, preventable risk factors, physical activity, obesity, smoking

## Abstract

The risk factors associated with metabolic syndrome (Met-S) including hypertension, hyperglycemia, central obesity, and dyslipidemia are preventable, particularly at their early stage. There are limited data available on the association between Met-S and preventable risk factors in young adults. We randomly selected 2,010 Saudis aged 18–30 years, who applied to be recruited in military colleges. All the procedures followed the guidelines of International Diabetes Federation. The results showed that out of 2,010 subjects, 4088 were affected with Met-S. The commonest risk factors were high blood sugar (63.6%), high systolic and diastolic blood pressures (63.3 and 37.3%), and high body mass index (57.5%). The prevalence of prediabetes and diabetes were 55.2 and 8.4%, respectively. Obesity, diabetes, hypertension, and hypertriglyceridemia were significantly associated with Met-S. The frequency of smoking was significantly linked with the development of Met-S. The prevalence of Met-S was found to be significantly higher in individuals with sedentary lifestyle. In conclusion, the results of this study clearly indicate that military recruits, who represent healthy young adults, are also prone to Met-S. The findings of this study will help in designing preventive measures as well as public awareness programs for controlling the high prevalence of Met-S in young adults.

## 1 Introduction

Metabolic syndrome (Met-S) is a major risk factor for cardiovascular disease (CVD) [1] and type-2 diabetes [2]. This syndrome is defined as a cluster of risk factors that typically include central obesity, elevated blood pressure (BP), impaired glucose metabolism, and dyslipidemia. In recent decades, marked socioeconomic developments in health, education, environment, and lifestyle in many developed countries have led to a decrease in communicable diseases, but an increase in chronic diseases of lifestyle, such as obesity, diabetes, hypertension, and other risk factors of CVD [3]. There are multiple risk factors associated with CVD such as behavioral factors (smoking, diet, physical activity [PA], alcohol consumption), physiological factors (blood cholesterol, hypertension, blood glucose, body mass index [BMI]), and metabolic disorders [4]. However, inadequate nutrient intake and low socioeconomic status are also linked with an elevated CVD risk [5,6].

Although the primary manifestations of CVD are common in older adults, they have also been detected in young adulthood [7,8]. Therefore, it is important to identify CVD risk factors in young persons with metabolic abnormalities with high risk of progression, as almost 50% of middle-aged men have abnormal glucose tolerance [9]. The obesity risk factors, such as unhealthy diet, physical inactivity, and sedentary behavior have been observed among adolescents; however, the association of these factors with obesity is not yet completely characterized [10,11]. Adolescents performing vigorous PA tend to consume a healthier diet and fewer unhealthy food items [11,12]. Healthy diet, active lifestyle as well as better cardiorespiratory fitness in adolescence have been associated with a reduced risk of CVD [13,14]. Lifestyle interventions including dietary modifications and increased PA play a significant role in the treatment of the obesity and related disorders such as impaired glucose intolerance, type 2-diabetes, and hyperlipidemia [9,11]. Increased PA in the intervention studies has resulted in beneficial changes in body composition, by reducing the amount of total and visceral fats, without a significant weight loss [9,11]. Many adolescents do not meet the health-related recommendations for sufficient PA, and the decline in PA has been observed from adolescence to young adulthood [15].

In fact, by identifying persons at risk of developing CVD and supplying early health counseling and lifestyle interventions, it could be possible to prevent later detrimental cardio-metabolic diseases. The unhealthy change in dietary habits, a sedentary lifestyle, and consanguineous marriages make the young Saudi population vulnerable to Met-S. The influence of diet, PA, and BMI on the body composition of adolescents and young adults has been studied previously [8,9,11]. However, there are limited data about the role of preventable risk factors for the development of Met-S in young adults, particularly in military personnel. Therefore, we investigated the status of Met-S in young Saudis enrolled for military recruitment. We specifically studied the association between Met-S and preventable risk factors including the body weight, PA, smoking, and dietary habits.

## 2 Materials and methods

This study was conducted on a total of 2,010 young Saudi men, aged 18–30 years, who applied for recruitment to Saudi armed forces. The study was carried out at the health facility of the selection centers and all the selected participants individually completed a consent form. Standardized medical observations included physical examination as well as measurements related to Met-S including BP, height, body weight, and blood biochemistry (blood glucose and lipid profile). The complete information of each participant was filled in a specially designed questionnaire based on the guidelines of the World Health Organization (WHO) [3]. The study protocol was approved (REC/523, dated 21/03/2017) by Institutional Ethical Committee.

According to the International Diabetes Federation (IDF) definition, subjects were considered to have Met-S if they had central obesity (defined as waist circumference >94 cm), plus two of the following four factors. Raised fasting plasma glucose >100 mg/dL (5.6 mmol/L), or previously diagnosed type-2 diabetes; systolic BP >130 mm Hg or diastolic BP >85 mm Hg, or treatment of previously diagnosed hypertension; high density lipoproteins (HDL) <40 mg/dL (1.0 mmol/L) or specific treatment for this lipid abnormality; and triglycerides (TGs) level >150 mg/dL (1.7 mmol/L) or specific treatment for this lipid abnormality.

Prehypertension was defined as systolic BP 120–139 mm Hg or diastolic BP 80–89 mm Hg. Hypertension was defined as systolic BP ≥140 mm Hg or diastolic BP ≥90 mm Hg [16]. BMI was classified according to the WHO adult BMI classification as normal (18.50–24.99 kg/m^2^), overweight (≥25–29.99 kg/m^2^), and obese (≥30 kg/m^2^) (Global Database on Body Mass Index: BMI classification [3]).

Blood samples from each recruitment center were transported to Prince Sultan Military Medical City for biochemical analysis. Blood samples were centrifuged at 1,500×*g* for 15 min, at 4°C, and sera were stored for analysis. Fasting blood sugar (FBS), total cholesterol, HDL, and TGs were analyzed using a Hitachi 902 autoanalyzer (Roche, Mannheim, Germany).

The data were analyzed by using the statistical package for the social sciences (SPSS) statistical package version 14 (SPSS Chicago, IL). Mean and standard deviation were calculated for parametric data, whereas categorical data were represented by number and percentage. The chi-square test and student *t*-test were used for comparison between the Met-S and without Met-S groups. Analysis of covariance with age-adjusted means was used to evaluate the association between Met-S component factors and different parameters. A two-tailed *P* value <0.05 was considered as statistically significant.

## 3 Results

### 3.1 Association between demography and Met-S

The impact of demographic characteristics including age, education, marital status, and monthly income on the development of Met-S is shown in Table 1. There was a direct association between age and Met-S. Younger subjects had significantly less frequency of Met-S as compared to older subjects (*P* < 0.001). The prevalence of Met-S was higher in subjects with primary education than those with secondary education (*P* < 0.001). Married subjects showed high frequency of Met-S as compared to unmarried participants (*P* < 0.01). Subjects coming from large families (>15 members) had significantly higher prevalence of Met-S (*P* < 0.05). Monthly income did not show any association with Met-S (Table 1).

**Table 1:** Association between Met-S and demographic characteristics

Demographic characteristics	Met-S		Total, *N*	*P* value
	Yes	No		
Age (years)				
≤21	283	1,165	1,448	0.000
22–26	182	331	513	
>26	23	26	49	
Total	488	1,522	2,010	
Education (years of study)				
≤14	287	1,183	1,470	0.000
15–19	199	334	533	
>19	2	5	7	
Total	488	1,522	2,010	
Marital status				
Married	31	46	77	0.003
Single	457	1,475	1,932	
Divorced	0	1	1	
Total	488	1,522	2,010	
Members in family <18 years				
≤5	287	972	1,259	0.039
6–10	153	435	588	
11–15	38	103	141	
>15	10	12	22	
Total	488	1,522	2,010	
Monthly income (Riyals)				
10,000	246	731	977	0.761
11,000–20,000	195	648	843	
>20,000	33	104	137	
Refused to answer	14	39	53	
Total	488	1,522	2,010	

### 3.2 Association between component factors and Met-S

We also analyzed the association between Met-S and the individual components that are used in the triplets of diagnosing Met-S. There was a direct relationship between bodyweight and Met-S. Individuals with the BMI <25 kg/m^2^ were free from Met-S, whereas overweight (40.26%) and obese (42.87%) subjects showed significantly high incidences of Met-S (Table 2). Subjects with hypertension also had significantly high (*P* < 0.001) frequency of Met-S as compared to subjects with normal BP. There was a direct association between FBS and Met-S. The prevalence of Met-S was highest in diabetic subjects (42.6%) followed by prediabetics (32.34%) as compared to subjects with normal FBS (7.79%; Figure 2). There was a direct correlation between TGs and Met-S, whereas an inverse correlation was observed between HDL and Met-S. Both these associations were statistically significant (*P* < 0.001) and of the same magnitude (Table 2).

**Table 2:** Association between Met-S and its individual component factors in subjects using the common cut-off values

Component factors	Met-S		Total, *N*	*P* value
	Yes	No		
BMI (kg/m^2^)				
≤18.4 (Underweight)	0	574	574	0.000
18.5–24.9 (Normal weight)	0	281	281	
25.0–29.9 (Overweight)	91	135	226	
≥30.0 (Obese)	397	532	929	
Total	488	1,522	2,010	
Systolic BP				
≤129 (Normal)	40	674	714	0.000
≥130 (High)	448	848	1,296	
Total	488	1,522	2,010	
Diastolic BP				
≤84 (Normal)	152	1,228	1,380	0.000
>84 (High)	336	294	630	
Total	488	1,522	2,010	
FBS (mg/dL)				
<100 (Normal)	57	674	731	0.000
100.0–125.9 (Prediabetic)	359	751	1,110	
≥126 (Diabetic)	72	97	169	
Total	488	1,522	2,010	
TGs (mg/dL)				
≤149.0 (Normal)	282	1,340	1,622	0.000
>149.0 (High)	206	182	388	
Total	488	1,522	2,010	
HDL (mg/dL)				
≤40.0 (Low)	127	108	235	0.000
>40.0 (Normal)	361	1,414	1,775	
Total	488	1,522	2,010	

### 3.3 Association between smoking habits and Met-S

Out of total 2,010 participants, only 94 (4.67%) were smokers. We observed a significant association between type of tobacco and Met-S (Figure 1). Age at start of smoking also played an important role in the progression of Met-S, as the current smokers showed significantly high frequency of Met-S. Previous history of smoking resulted in significantly high frequency of Met-S (*P* = 0.005), whereas an early cessation of smoking significantly reduced the incidence of Met-S (*P* = 0.002). Although the use of smoke-less tobacco (SLT) was not associated with Met-S, the rate of consuming SLT showed a significant direct association with Met-S (*P* = 0.001). Passive smoking was reported by 14% subjects; however, there was no significant association between passive smoking and Met-S (Figure 1).

**Figure 1:** Association between Met-S and smoking habits or use of tobacco. Values are percentage frequency of Me-S in the same category.

### 3.4 Association between dietary habits and Met-S

Fruit and vegetable consumptions per se were not associated (*P* = 0.411 for fruits and *P* = 0.435 for vegetables) with the prevalence of Met-S in subjects (Table 3). Type of cooking oil and eating fast foods were also not associated with Met-S in young adults (Table 3).

**Table 3:** Association of Met-S with feeding habits and nutrition

Feeding and nutrition	Met-S		Total, *N*		
	Yes	No		*P* value	
Do you eat fruits					
Yes	410	1,287	1,697		0.411
No	78	235	313		
Total	488	1,522	2,010		
Fruits consumption (FC)/week					
No fruit consumption/week	71	205	276		0.025
1.0–3.0 (Times/week)	277	974	1,251		
4.0–6.0 (Times/week)	69	164	233		
>6.0 (Times/week)	71	179	250		
Total	488	1,522	2,010		
FC/day					
No fruit consumption/day	71	205	276		0.166
1.0–3.0 (Times/day)	414	1,306	1,720		
4.0–6.0 (Times/day)	0	8	8		
>6.0 (Times/day)	3	3	6		
Total	488	1,522	2,010		
Do you consume vegetables?					
Yes	446	1,385	1,831		0.435
No	42	137	179		
Total	488	1,522	2,010		
Veg/week					
No vegetable consumption	34	108	142		0.288
1.0–3.0 (Times/week)	161	541	702		
4.0–6.0 (Times/week)	92	232	324		
>6.0 (Times/week)	201	641	842		
Total	488	1,522	2,010		
Veg/day					
No veg. consumption/day	42	137	179		0.992
1.0 (Once per day)	382	1,187	1,569		
2.0 (Twice per day)	51	156	207		
>2.0 (More times/day)	13	42	55		
Total	488	1,522	2,010		
Type of cooking oil					
Non-user	9	38	47		0.108
Veg. oil	395	1,228	1,623		
Veg. fat	0	10	10		
Butter	2	0	2		
Animal fat	5	6	11		
Veg. oil and veg. fat	15	49	64		
Veg. oil and butter	7	18	25		
Veg. oil and animal fat	34	98	132		
Veg. oil, veg. fat, and butter	0	3	3		
Veg. oil, veg. fat, and anim. fat	2	9	11		
Veg. oil, butter, and anim. fat	19	55	74		
Veg. oil, veg. fat, butter, and anim. fat	0	8	8		
Total	488	1,522	2,010		
Eating fast food					
Yes	420	1,313	1,733		0.481
No	68	209	277		
Total	488	1,522	2,010		
If yes eating-time?					
Not eating fast food	68	209	277		0.562
Breakfast	19	43	62		
Lunch	32	71	103		
Dinner	203	655	858		
Breakfast and lunch	2	3	5		
Breakfast and dinner	81	252	333		
Lunch and dinner	59	213	272		
Breakfast, lunch, and dinner	24	76	100		
Total	488	1,522	2,010		
Days/week					
Not eating fast food	68	209	277		0.130
1–3 (Days/week)	270	792	1,062		
4–6 (Days/week)	99	298	397		
7 (Days/week)	51	223	274		
Total	488	1,522	2,010		

### 3.5 Association between PA and Met-S

A simple query about PA (Yes or No) did not reveal any association between PA and Met-S (*P* = 0.263; Table 4). However, a categorical breakup of data about the preferences of subjects for footing or driving for various activities including work, prayer, shopping, or combination of these activities showed significant association between mode of PA and Met-S (Table 4).

**Table 4:** Association between Met-S and PA

PA	Met-S		Total, *N*	*P* value
	Yes	No		
PA				
Yes	433	1,377	1,810	0.263
No	55	145	200	
Total	488	1,522	2,010	
By foot				
No footing	55	140	195	0.000
Work (footing)	5	16	21	
Prayer (footing)	286	758	1,044	
Shopping (footing)	6	19	25	
Work and prayer (footing)	16	38	54	
Work and shopping (footing)	0	5	5	
Prayer and shopping (footing)	88	462	550	
Work, prayer, shopping (footing)	32	84	116	
Total	488	1,522	2,010	
By car				
Work (Driving)	84	351	435	0.026
Prayer (Driving)	9	16	25	
Shopping (Driving)	120	298	418	
Work and prayer (Driving)	2	3	5	
Work and shopping (Driving)	173	574	747	
Prayer and shopping (Driving)	50	146	196	
Work, prayer, shopping (Driving)	50	134	184	
Total	488	1,522	2,010	
By foot/week				
None	55	140	195	0.187
1–3 Days	5	20	25	
4–6 Days	4	30	34	
7 Days	424	1,332	1,756	
Total	488	1,522	2,010	
By car/week				
Up to 3 days	19	63	82	0.523
4–6 Days	78	276	354	
7 Days	391	1,183	1,574	
Total	488	1,522	2,010	
Time spent driving car/day in minutes				
Up to 100 min	227	731	958	0.160
101–200 min	134	467	601	
201–300 min	89	228	317	
>300 min	38	96	134	
Total	488	1,522	2,010	
Time spent on foot/day in minutes				
No footing period	55	140	195	0.293
<30 min	282	883	1,165	
31–60 min	93	277	370	
>60 min	58	222	280	
Total	488	1,522	2,010	

### 3.6 Association between recreational activity and Met-S

The participants who used to be involved in recreational activity had significantly less frequency of Met-S (*P* = 0.042; Figure 2). Those who were involved in rigorous intensive sports showed significantly decreased occurrence of Met-S (*P* < 0.001). Moreover, the time spent is rigorous sporting activity also showed a significant association with Met-S (Figure 2). There was no significant difference in the prevalence of Met-S among those subjects who were involved in moderate physical activity (MPA) compared to those who were not involved in MPA (Figure 3). Even the regularity in MPA was not significantly associated with the incidence of Met-S (Figure 3).

**Figure 2:** Association between vigorous intensive sports and Met-S. Values are percentage frequency of Met-S in the same category.

**Figure 3:** Association between MPA and Met-S. Values are percentage frequency of Met-S in the same category.

## 4 Discussion

Our results showed that demographic factors including age, education level, marital status, and family size are significantly associated with Met-S; however, monthly income did not show any association with Met-S (Table 1). All the component factors including BMI, BP, blood sugar, TGs, and HDL showed highly significant (*P* < 0.001) association with Met-S (Table 2). A direct correlation of age with Met-S has also been reported by previous investigators [17,18]. Alexander et al. [19] reported that blood glucose, diabetes and BP had a direct relationship with age and BMI, and that prevalence of diabetes and hypertension (components of Met-S) increased with age, which also increased the incidence of Met-S. It has been shown that alarming rates of some risk factors increase with age in cases of diabetes, hypertension, and obesity, and they could be attributed to uncontrolled hyperglycemia and reduced PA in older individuals [8,20].

In our study on young adults, the prevalence of diabetes was found to be 8.40% (Table 2). According to 2014 data, more than 20% of the Saudi Arabian adult population has diabetes while the total number of undiagnosed cases of diabetes among adults is estimated to be more than 1.5 million [21,22]. The projected trajectory for diabetes in Saudi Arabia is alarming, particularly among the 40–49 age group [21]. The increase in the incidence of diabetes in Saudi Arabia has been attributed to changes in cultural and socioeconomic factors, such as increase in affluence, physical inactivity, and changes in dietary habits with the substitution of animal products and refined foods [23,24].

We also observed high prevalence of overweight (11.24%) and obesity (46.21%) in our study population (Table 2). The high rate of overweight and obesity among adolescents is a major public health problem in Saudi Arabia, and is growing at an alarming rate [25], which is more prevalent in Saudi women than in men [26]. Even high frequencies of overweight (15.5%) and obese (6%) have been reported in Saudi schoolchildren [27]. A survey conducted in 2015 among schoolchildren in Riyadh city showed the overall prevalence of overweight and obesity as 13.4 and 18.2%, respectively [28]. In a survey conducted in 2013, the prevalence of obesity was higher among Saudi women (33.5 versus 24.1%), and obesity was strongly associated with diabetes, hypercholesterolemia, hypertension, marital status, and PA [29]. In a later study, the overall prevalence of overweight and obesity among adults visiting primary care settings in the Southwestern Region of Saudi Arabia was found to be 38.3 and 27.6%, respectively [30]. Mosli et al. [31] observed that individuals in the highest income bracket with lower levels of education have greater odds of obesity. The prevalence of obesity among adults in Saudi Arabia increased from 22% in 1990–1993 to 36% in 2005, and future projections of the prevalence of adult obesity in 2022 was estimated to be 41% in men and 78% in women [32]. Thus, the prevalence of obesity found in our study is comparable to earlier predictions. Military recruits are now less physically fit and more massive, with elevated body fat, highlighting the necessity for regular surveys, monitoring, and effective primary prevention strategies [33]. Obesity is a progressively significant public health problem and is considered a major risk factor for diet-related chronic diseases including Met-S, diabetes, hypertension, stroke, and certain forms of cancer [34].

Although we did not observe a significant association between intake of fruit and vegetables (F&V) and Met-S (Table 3), it has shown beneficial effects on related ailments. A study on 65,226 subjects found that daily eating ≥7 portions of F&V reduced the risk of death due to heart disease by 31% [35]. The Physicians’ Health Study, during a follow-up of 12 years, reported 25% lower incidence of coronary artery disease (CAD) in men who consumed >2.5 or more serving of vegetables daily, compared with those who consumed less than one serving daily [36]. It has been shown that diets high in fiber are significantly associated with lower risks of CVD (stroke and CAD) [37]. Another large prospective cohort study of 84,251 women in the Nurse’ Health Study and 42,148 men in the Health Professionals Follow-up Study reported 30% lower risk of CVD in people with high F&V intake (more than five serving daily) compared to those with low intake. For each increase of one serving per day in F&V, a 4% lower risk of coronary heart disease and 6% lower risk of ischemic stroke were observed [38].

In this study, the mode of tobacco use was significantly associated with Met-S (Figure 1). The global adult tobacco survey showed that in nine Arab countries (Bahrain, Egypt, Libya, Jordan, Kuwait, Lebanon, Palestine, Tunisia, and Syria), the prevalence of daily tobacco use exceeds 30% in men [39]. Water pipe smoking is increasing in young Arabs with prevalence estimates between 6 and 34% in age group of 13–15 years [40]. Azadbakht et al. [41] reported that avoiding smoking and limiting alcohol could be beneficial in reducing most of the metabolic risk factors in both sexes. Cigarette smoking increases inflammation and thrombosis leading to oxidative stress manifestation, prothrombotic activity, platelet aggregation, leukocyte activation, lipids peroxidation, and smooth muscle proliferation [42]. Nicotine affects the cardiovascular system by increasing systolic and diastolic BP, heart rate, and cardiac output [43].

We observed a significant role of PA in the development of Met-S. A high prevalence (70%) of physical inactivity has been reported in individuals from gulf countries [39]. Potential influences on individual’s lifestyle were affected by the economic transition in Saudi Arabia through the contribution expedited by recent patterns in occupations that offered inadequate physical activities [8,44]. Physical inactivity is a predictor of CVD events and associated mortality. Sedentary lifestyle for a longer period leads to Met-S and its components, such as increased adipose tissue (predominantly central), reduced HDL cholesterol and a trend towards increased TGs and glucose in genetically susceptible persons. Individuals who spend more than 4 h/day watching television or videos or use their computers have a two-fold increased risk of Met-S compared to those who spend less than 1 h [45].

It is important to note that many risk factors become more damaging when they occur in combination with one another. Most of these risk factors are avoidable and can easily be managed by lifestyle changes. Modifiable risk factors, including hypertension, smoking, diabetes, obesity, dyslipedemia, stress, unhealthy diet, and physical inactivity, are the major contributors to cardiovascular morbidity and mortality. These risk factors rarely occur alone, and instead tend to cluster in individuals [46]. The prevalence of uncontrolled hyperglycemia was reported to be high among Saudi diabetic patients while the associated risk factors included older age, male gender, hypertension, smoking, and obesity [47]. Moreover, uncontrolled hyperglycemia has also been directly associated with dyslipidemia [48,49]. It has been demonstrated that five modifiable risk factors such as cigarette smoking, overweight or obesity, hypertension, diabetes, and dyslipidemia can be eliminated by management [11]. The occurrence of multiple risk factors is more common, which increases the individual’s risk of CVD from 4-fold with one risk factor to 60-fold in the cluster of five risk factors [50]. The prevalence of multimorbidity (two or more chronic conditions) is increasing, due to growing incidence of chronic conditions and increasing life expectancy [51]. The global burden disease for risk profiles in Middle East and North Africa stranded out these risk factors by order of priority: high BP ranked as the first, followed by obesity, diabetes, smoking, and dyslipidemia [52]. Met-S is progressive, and early indications of disease are evident in adolescents and young adults [53,54]. Some reports suggest that a large number of adolescents already carry one or more risk factors for Met-S [55,56]. Exposure to Met-S risk factors in childhood and adolescence is associated with disease development in adulthood [57,58]. Health risk behaviors tend to establish quite early in life; identifying strategies that deter the adoption and continuation of these health risk factors in younger adults is essential for a long-term prevention of Met-S.

In conclusion, Met-S is prevalent in young military recruits, which is a matter of great concern. Several demographic factors such as age, education, marital status, and family size were significantly associated with Met-S. The component factors of Met-S including BMI, BP, blood sugar, TGs, and HDL showed highly significant association with Met-S. Most of these factors are preventable and can be controlled by modifications in dietary habits and PA. Although MPA was not very effective in reducing Met-S, rigorous physical work and sport activities significantly reduced the incidence of Met-S. These findings will help in designing preventive measures as well as public awareness programs for controlling the high prevalence of Met-S in young adults.
